# Clinical Effect of Nicorandil Combined with Aspirin in the Treatment of Myocardial Ischemia

**DOI:** 10.1155/2022/2214411

**Published:** 2022-05-18

**Authors:** Yue Li, Chen Zhao, Chengxin Xiong, Yuping Gao

**Affiliations:** ^1^Department of Cardiology, Third Hospital of Shanxi Medical University, Key Laboratory of Cellular Physiology (Shanxi Medical University), Ministry of Education, China; ^2^School of Computer Science, Hefei University of Technology, China

## Abstract

**Objective:**

To investigate the clinical effect of nicorandil combined with aspirin in the treatment of myocardial ischemia.

**Methods:**

A total of 104 patients with myocardial ischemia were admitted to our hospital from June 2019 to August 2020. These patients were selected as the research objects and randomly divided into two groups: the control group and the observation group. The control group was given asilin, and the observation group was given nicorandil tablets based on the control group. Both groups were given continuous treatment for 3 months. The curative effect, cardiac function indexes, dynamic electrocardiogram, and the occurrence of adverse reactions were observed in the two groups.

**Results:**

The total effective rate of the observation group was 96.15% (50/52), which was higher than that of the control group (61.54%, 32/52), and the difference was statistically significant (*P* < 0.05). After treatment, left ventricular ejection fraction (LVEF) and peak early/late diastolic flow velocity (E/A) were increased (*P* < 0.05), while peak early diastolic flow velocity to peak mitral annular root movement velocity (E/Ea) was decreased (*P* < 0.05). After treatment, LVEF and E/A in the observation group were higher than those in the control group, while E/Ea was lower than that in the control group (*P* < 0.05). The frequency, duration of ST segment, and a total load of myocardial ischemia in the ST segment within 24 h after treatment were decreased compared with those before treatment (*P* < 0.05). The frequency and duration of ST segment decreased, and the total load of myocardial ischemia in the observation group was lower than those in the control group within 24 h after treatment (*P* < 0.05). After treatment, the total occurrence of adverse reactions in the observation group was lower than that in the control group (*P* < 0.05).

**Conclusion:**

Nicorandil combined with aspirin in the treatment of patients with myocardial ischemia has a significant effect, which can effectively improve the electrocardiogram and cardiac function indicators of patients and reduce the incidence of adverse reactions and is worthy of clinical application.

## 1. Introduction

The continuous change of dietary structure and the increasing pressure of life are one of the important factors for the increase of the number of patients with hypertension. These changes have promoted chronic coronary endothelial injury and coronary artery stenosis caused by primary hypertension and hyperlipidemia, which led to the occurrence of myocardial ischemia in patients [1, 2]. Clinically, there are many reasons for myocardial ischemia, including an inability to remove metabolites, myocardial hypoxia, and decreased coronary blood flow [3]. Myocardial ischemia can cause myocardial infarction in patients, and some patients may die of sudden death, which seriously threatens the life safety of patients [4]. Myocardial ischemia is one of the common diseases of coronary heart disease. At the onset of this disease, patients with myocardial activity and metabolism have different degrees of abnormal changes, resulting in cardiac function changes and arrhythmia [5, 6]. Currently, aspirin is mainly used to treat this disease clinically, which reduces blood viscosity by inhibiting the generation of platelets [7]. Nicorandil can act on coronary arteries and vessels to improve myocardial ischemia. The combination of nicorandil and aspirin can enhance the clinical effect of treating myocardial ischemia [8]. Nicorandil belongs to the adenosine triphosphate K+ channel opening agent and has the effect of dilating coronary artery, relieving coronary spasms, and increasing myocardial blood supply [9]. According to the study, nicorandil has the function of diastolic blood vessels, increasing coronary blood flow, and is mostly used in the treatment of myocardial ischemia [10]. Based on this, 104 cases of patients with myocardial ischemia admitted to our hospital from June 2019 to August 2020 were selected as the research objects to explore the clinical effect of nicorandil combined with aspirin in the treatment of patients with myocardial ischemia. The specific contents are reported as follows.

The major contributions of this paper are given below:

- In this paper, the researchers have analyzed the clinical effect of nicorandil combined with aspirin in the treatment of patients with myocardial ischemia
- A total of 104 patients with myocardial ischemia admitted were divided into two groups: (i) the control group and (ii) the observational group
- The control group was treated with asilin, while the observational group was treated with nicorandil tablet
- The comparison of curative effects, cardiac function indexes in LVEF, E/A, and E/Ea, comparison of dynamic electrocardiogram, and comparison of the occurrence of adverse reactions between the two groups before and after the treatment were assessed
- Research in this study showed that nicorandil combined with aspirin in the treatment of patients with myocardial ischemia has a significant effect. After treatment, the obvious effect was that the symptoms disappeared and the heart function improved to a significant level

The outline of this paper is given below.

In Section 1, the general information of the patients has been collected in the hospital and treated with general treatment. Patients with myocardial ischemia are collected and divided into the control group and the observation group. The control group was treated with asilin, while the observational group was treated with nicorandil tablet.

In Section 2, the results of curative effects, comparison of cardiac function indexes in LVEF, E/A, and E/Ea, comparison of dynamic electrocardiogram, and comparison of the occurrence of adverse reactions between the two groups before and after the treatment are obtained.

In Section 3, treatment for myocardial ischemia in patients has been discussed. After treatment, the symptoms disappeared and the heart function improved to a significant level. The heart function of the two groups of patients was significantly improved compared with before the treatment.

In the end, it is concluded that nicorandil combined with aspirin in the treatment of patients with myocardial ischemia has improved to a significant level significant effect.

## 2. Material and Methods

In this section, the general information of the selected patients with myocardial ischemia is collected and divided into the control group and the observation group. Treatment for the patients in the control group and observation group is discussed. The observation index, treatment effectiveness, and statistical analysis are discussed.

### 2.1. General Information

A total of 104 patients with myocardial ischemia admitted to our hospital from June 2019 to August 2020 were selected as the research objects and randomly divided into control group and observation group, with 52 cases in each group.

Inclusion criteria were as follows: myocardial ischemia was confirmed by coronary angiography in all patients. Patients for the treatment must have systolic pressure < 90 mm Hg. Patients before the treatment should not take other types of drugs to improve myocardial perfusion. All patients were informed of this study and had signed informed consent before the treatment. Before the treatment, complete clinical data should be collected from the patient.

Exclusion criteria were as follows: with severe abnormal liver and kidney function, mental illness, pregnant or breastfeeding women, allergic, and those who used other related drugs within 1 week before treatment.

There was no significant difference in general data between the two groups (*P* > 0.05), indicating comparability. With the approval of the Ethics Committee of our school, general information about the two groups is shown in Table 1.

### 2.2. Methods

Both groups received symptomatic treatment and basic treatment according to the symptoms of chest distress, shortness of breath, palpitation, and other symptoms in each group.

- Control group received aspirin (national drug approval H44021505; Produced by Shantou Jinshi Pharmaceutical General Factory Co., LTD). The approved control group would be administered after no history of allergies. The initial dose was 50 mg. For objects with severe illness, the administration would be 100 mg. The poorly tolerated objects were given two doses of 25 mg each time. The continuous medication for 7 days constituted a course of treatment, and a total of four courses of treatment were given
- Observation group was given nicorandil tablet (Liaoyuan Baikang Pharmaceutical Co., Ltd., 5 mg/tablet) 1 tablet each time, 3 times a day, based on the control group. Patients in both groups took the drug continuously for 3 months

### 2.3. Observation Index

The treatment time of the two groups was 3 months, and the outcome indexes of the two groups were compared, including curative effect, cardiac function indexes, dynamic electrocardiogram, and the occurrence of adverse reactions.

#### 2.3.1. Curative Effect

Efficacy criteria were as follows: significant effects were found after treatment, the main symptoms disappeared, and the myocardial ischemia load and ST segment depression times were significantly improved. The effectiveness of treatment can be found after the main symptoms were improved, and the number of myocardial ischemia load and ST segment depression was improved. Ineffectiveness: there was no improvement in major symptoms, myocardial ischemic load, and frequency of ST segment depression. Obvious and effective add up to total effectiveness.

#### 2.3.2. Cardiac Function Indexes

The left ventricular ejection fraction (LVEF), peak early/late diastolic flow velocity (E/A), and the ratio of peak early diastolic flow velocity to peak mitral annular root movement velocity (E/Ea) before and after treatment were examined by IE-33 color Doppler ultrasonography (Philips) to assess cardiac function [11].

#### 2.3.3. Dynamic Electrocardiogram

Dynamic electrocardiogram was performed before and after treatment to compare the frequency and duration of ST segment decline within 24 h between the two groups, and the total myocardial ischemia load was calculated. Total myocardial ischemia load = ST segment depression (mm) × duration (min) [12].

#### 2.3.4. Occurrence of Adverse Reactions

These included low headache, angina, hypotension, palpitations, and arrhythmias.

### 2.4. Efficacy Criteria

The obvious effect was that the symptoms disappeared and the heart function improved to a significant level. Effective symptom improvement means heart function improved; ineffectiveness means no significant change, aggravation, or death in cardiac function. Total effective rate (%) = (number of effective cases + number of effective cases)/total number of cases × 100%.

### 2.5. Statistical Method

SPSS 21.0 software was used to statistically analyze the data of patients in the two groups. A *t*-test was used to measure data as (*x* ± *s*), a *χ*^2^ test was used to count data as (%), and *P* < 0.05 was used to indicate that the difference was statistically significant.

## 3. Results

In this section, the comparison of curative effects, comparison of cardiac function indexes in LVEF, E/A, and E/Ea, comparison of dynamic electrocardiogram, and comparison of the occurrence of adverse reactions between the two groups before and after the treatment are discussed.

### 3.1. Comparison of Curative Effect between Two Groups

The total effective rate of the observation group was 96.15% (50/52), which was higher than that of the control group (61.54%, 32/52), and the difference was statistically significant (*P* < 0.05). A comparison of the curative effect between the two groups is shown in Table 2.

### 3.2. Comparison of Cardiac Function Indexes before and after Treatment

There were no significant differences in LVEF, E/A, and E/Ea between the two groups before treatment (*P* > 0.05). After treatment, LVEF and E/A were increased (*P* < 0.05), while E/Ea was decreased (*P* < 0.05). After treatment, LVEF and E/A in the observation group were higher than those in the control group, while E/Ea was lower than that in the control group (*P* < 0.05). A comparison of cardiac function indexes before and after treatment is shown in Table 3.

### 3.3. Comparison of Dynamic Electrocardiogram between the Two Groups before and after Treatment

There were no significant differences in the frequency, duration of ST segment, and total load of myocardial ischemia in the two groups within 24 h before treatment (*P* > 0.05), while the frequency, duration of ST segment, and total load of myocardial ischemia in the ST segment within 24 h after treatment were decreased compared with those before treatment (*P* < 0.05). The frequency and duration of ST segment decreased, and total load of myocardial ischemia in the observation group was lower than those in the control group within 24 h after treatment (*P* < 0.05). A comparison of dynamic electrocardiogram between the two groups before and after treatment is shown in Table 4.

### 3.4. Comparison of Occurrence of Adverse Reactions between the Two Groups

After treatment, the total occurrence of adverse reactions in the observation group was lower than that in the control group (*P* < 0.05). A comparison of the occurrence of adverse reactions between the two groups was shown in Table 5.

## 4. Discussion

Myocardial ischemia is a pathological state in which the blood perfusion to the heart is abnormal, affecting cardiac function, limiting blood supply, and affecting cardiac energy metabolism and overall function in a relatively short time [13]. This disease has an urgent onset, complicated etiology, and the possibility of death, which puts forward high requirements for treatment [14, 15]. When the symptoms of myocardial ischemia occur, the coronary artery blood flow in the patient's body is continuously reduced, resulting in the continuous weakening of the metabolic capacity in the patient's body, and then, hypoxia occurs [16]. In the past, aspirin was widely used in clinical treatment, which could alleviate the myocardial ischemia symptoms of patients to a certain extent, but the effect was not obvious [17]. The study found that the addition of nicorandil to aspirin could further dilate the blood vessels, thus enhancing the efficacy of the treatment [18, 19]. Among them, nicorandil is a nitro-based compound, which has the effect of dilating the vascular smooth muscle of the circulatory system, and its pharmacological effect is similar to that of nitrate drugs. Nicorandil has a significant coronary artery dilating effect, which can increase the blood flow at the site of coronary artery stenosis and increase the oxygen supply of ischemic myocardium [20]. At the same time, it can also act on the K+ channel of the myocardial cell membrane, increase the K+ inflow, reduce the Ca2+ inflow, reduce the Ca2+ overload in ischemic cardiomyocytes, protect vascular endothelial cells, reduce the apoptosis of cardiomyocytes, and reduce the injury of cardiomyocytes [21].

The results of this study showed that the total effective rate of the observation group was 96.15% (50/52), which was higher than that of the control group (61.54%, 32/52), and the difference was statistically significant (*P* < 0.05). After treatment, LVEF and E/A were increased (*P* < 0.05), while E/Ea was decreased (*P* < 0.05). After treatment, LVEF and E/A in the observation group were higher than those in the control group, while E/Ea was lower than that in the control group (*P* < 0.05). The frequency, duration of ST segment, and a total load of myocardial ischemia in the ST segment within 24 h after treatment were decreased compared with those before treatment (*P* < 0.05). The frequency and duration of ST segment decreased, and the total load of myocardial ischemia in the observation group was lower than those in the control group within 24 h after treatment (*P* < 0.05). After treatment, the total occurrence of adverse reactions in the observation group was lower than that in the control group (*P* < 0.05).

In conclusion, nicorandil combined with aspirin in the treatment of patients with myocardial ischemia has a significant effect, which can effectively improve the electrocardiogram and cardiac function indicators of patients and reduce the incidence of adverse reactions and is worthy of clinical application.

## Figures and Tables

**Table 1:** General information of two groups.

General information	Observation group	Control group	*P*
Cases	52	52	>0.05
Gender			
Male	29	27	>0.05
Female	23	25	
Age (average)	52.34 ± 9.53	50.65 ± 9.02	>0.05
Course of disease (average)(year)	4.36 ± 1.17	4.70 ± 0.83	>0.05

**Table 2:** Comparison of curative effect between two groups.

Groups	Cases	Significant effect	Effective	Ineffectiveness	Total effective rate
Observation group	52	22	28	2	50 (96.15%)
Control group	52	13	19	20	32 (61.54%)
*χ* ^2^		5.664	0.329	5.132	5.104
*P*		<0.05	<M0.05	<0.05	<0.05

**Table 3:** Comparison of cardiac function indexes before and after treatment.

Groups	Observation group	Control group	*t*	*P*
LVEF				
Before treatment	42.13 ± 5.03	42.06 ± 5.40	1.147	>0.05
After treatment	55.89 ± 6.94	50.11 ± 5.03	4.156	<0.05
E/A				
Before treatment	0.89 ± 0.11	0.86 ± 0.12	1.021	>0.05
After treatment	1.92 ± 0.24	1.30 ± 0.27	8.063	<0.05
E/Ea				
Before treatment	10.62 ± 2.39	10.54 ± 2.33	1.152	>0.05
After treatment	4.35 ± 0.88	7.12 ± 1.02	4.672	<0.05

**Table 4:** Comparison of dynamic electrocardiogram between the two groups before and after treatment.

Groups	Observation group	Control group	*t*	*P*
Frequency of ST segment (times)				
Before treatment	8.76 ± 1.23	8.59 ± 1.41	1.107	>0.05
After treatment	2.08 ± 0.76	4.59 ± 0.67	4.685	<0.05
Duration of ST segment (min)				
Before treatment	54.82 ± 8.16	54.08 ± 8.64	1.089	>0.05
After treatment	11.29 ± 2.61	28.67 ± 3.69	6.825	<0.05
Total load of myocardial ischemia (mm·min^−1^)				
Before treatment	98.84 ± 11.05	97.76 ± 10.53	1.246	>0.05
After treatment	21.55 ± 3.58	40.57 ± 4.16	8.050	<0.05

**Table 5:** Comparison of occurrence of adverse reactions between the two groups.

Groups	Low headache	Angina	Hypotension	Palpitations	Arrhythmias	Total occurrence rate
Observation group	0	2	1	1	0	7.69%
Control group	3	6	4	5	3	40.38%
*x* ^2^	7.825	2.018	0.604	7.005	0.218	13.824
*P*	<0.05	<0.05	<0.05	<0.05	<0.05	<0.05

## Data Availability

The data used to support the findings of this study are included within the article.
